# Renoprotective and Cardioprotective Potential of *Moricandia sinaica* (Boiss.) against Carbon Tetrachloride-Induced Toxicity in Rats

**DOI:** 10.1155/2022/8545695

**Published:** 2022-06-29

**Authors:** Abdelaaty A. Shahat, Heba D. Hassanein, Riaz Ullah, Ali S. Alqahtani, Husseiny A. Husseiny, Alicja Kowalczyk, Abdel-Razik H. Farrag

**Affiliations:** ^1^Department of Pharmacognosy, College of Pharmacy, King Saud University, Riyadh 11451, Saudi Arabia; ^2^Chemistry of Medicinal Plants Department, National Research Centre, 33 El Bohouth St. (Former El Tahrirst.), Dokki, P.O. 12622, Giza, Egypt; ^3^Faculty of Pharmacy, Misr University for Science and Technology (MUST), Giza, Egypt; ^4^Department of Environmental Hygiene and Animal Welfare, Wrocław University of Environmental and Life Sciences, Chełmońskiego 38C, Wrocław 51-630, Poland; ^5^Pathology Department, National Research Centre, 33 El Bohouth St. (Former El Tahrir St.), Dokki, P.O. 12622, Giza, Egypt

## Abstract

The goal of the current study was to assess the nephroprotective and cardioprotective potential of *Moricandia sinaica* methanol extract (MOR-1), as well as its butanol (MOR-2) and aqueous (MOR-3) fractions against carbon tetrachloride (CCl_4_)-induced nephro and cardio-toxicity. Cardiac function was assessed using the biochemical parameters lactate dehydrogenase (LDH) and creatinine kinase (CK). Renal function was examined using the biochemical parameters creatinine and uric acid. The levels of nonprotein sulfhydryls (NPSH) and malondialdehyde (MDA) were used as markers of oxidative strain. A dose of 100 and 200 mg/kg of butanol fraction given prior to CCl_4_ treatment significantly (*p* < 0.05 − 0.001) protected against elevated LDH and CK levels. Similarly, treatment with silymarin (10 mg/kg) and butanol fraction (100 and 200 mg/kg) significantly (*p* < 0.05 − 0.001) boosted total protein levels compared to CCl_4_ treatment alone. The silymarin (10 mg/kg) and butanol fraction (100 and 200 mg/kg) also provided a significant (*p* < 0.05 − 0.001) protective effect for MDA levels. Methanol extract (MOR-1) and butanol (MOR-2) showed significant results and were recommended for further pharmacological and screening for active constituents.

## 1. Introduction

Medicinal plants provide a wealth of primary and secondary metabolites, including carbohydrates, proteins, lipids, alkaloids, glycosides, tannins, and a variety of other compounds. Traditional medicine has historically relied on herbs and plants. Herbs are thought to be a treasure trove of phytochemicals with a diverse variety of pharmacological effects. The herbs that house these various elements are a natural gift. Alkaloids, flavonoids, and saponin are some of the secondary metabolites that have significant therapeutic value. Multiple chronic diseases, such as diabetes, cardiovascular disease, chronic fatigue syndrome, and a variety of infections, are treated as a result of the existence of such metabolites. Many scientific research have shown that these primary and secondary metabolites have the ability to treat a variety of acute and chronic disorders [1–3]. Several anticancer drugs, including vinblastine and paclitaxel, are exclusively derived from botanicals. Similarly, aspirin, a recognized pain killer, is actually a derivative of Salix and Spiraea species [4]. Concerning the extreme usage of botanical remedies as health care medications, it has developed an imperative stage to screen the medicinal plants for active phytoconstituents, which are the foundation for the search of cancer-related and antibiotic drugs [5]. Apparently, natural products will endure being tremendously imperative as the foundation of medicinal plant agents. [6]. Globally, the mainstream of the population practices traditional medicine for the treatment of their ailments. Floras are observed as valued foundations for the advancement of novel medications by several investigators. At present, herbal medicine is extensively practiced to avoid or switch the sicknesses and more than a few medicinal plants are being regularly investigated in relation to antiinflammatory, antiapoptotic, antibiotic, antimicrobials, antioxidants, anticancer, and other pharmacological activities [7].

Traditional medicinal plants as herbal drugs have become common due to their efficacy and safety for the heeling of cardiac and nephrotoxicity. In the last two decades, traditional medicine, particularly herbal treatments, has been increasingly popular. So, because markets for pharmaceuticals are quickly growing and significant economic gains are being generated, equally urbanized and upward countries are showing a great deal of interest in herbal medication plantation and rearing [8, 9]. Chemicals like polycyclic aromatic hydrocarbons, acetaminophen, CCl_4,_ etc., cause root tissue damage in animals as well as in humans. CCl_4_ is known for the initiation of the making of oxygen free radicals in various tissues such as the blood, brain, kidney, and liver. CCl_4_ is disintegrated into trichloromethyl peroxyl (Cl_3_COO**•**) and trichloromethyl (CCl_3_**•**) radicals by the cytochrome oxidase enzyme complex. These free radicals cause cytoplasmic membrane phospholipids to endure lipid peroxidation. Practical variations happen in the cell membrane as a consequence of the peroxidation of lipid [10]. CCl_4_ is a potent lipid-soluble hepatotoxin bound to lipid and protein, and is used to enhance the peroxidative process [11]. Its toxic effect is dependent on the excessive production of the trichloromethyl peroxyl radical (CCl_3_^•^) [12]. It can be the source of the development of reactive oxygen species (ROS) in various dynamic tissues such as the blood, brain, kidney, and liver [13]. Toxic free radicals lead to noticeable lipid peroxidation that results in disproportionate impairment to cell membranes and the growth of a number of pathological changes in renal damage [14]. These toxic renal effects occur via the destruction of renal mitochondrial function, including across mitochondrial membranes.

Numerous medicinal plants have been described to display care output of renal tissues against damage. Nephroprotective effects were mediated via modulating the expression of inflammatory, oxidative stress, and apoptotic mediators [15]. Some species from the Brassicaceae family have shown nephroprotective activity, such as the methanol extract of *Brassica nigra* leaves against D-galactosamine-induced nephrotoxicity, as well as, the ethanol extract of *Brassica rapa* roots against cisplatin-induced nephrotoxicity. *Moricandia sinaica* specie belongs to the family Brassicaceae, which has very few studies on its biological evaluation. Thus, the aim of this study is to evaluate the nephro and cardio protective effect of *Moricandia sinaica* against CCl_4_-induced toxicity [15, 16]. In our earlier investigation, 24 secondary metabolites were found in *Moricandia sinaica* using HPLC-MS/MS. The compounds included lucosinolates, phenolic acids, and flavonoids. Docking results discovered that polyphenols found delivered virtuous potent constituents for the development of safe and novel drugs agent [17].

## 2. Materials and Methods

### 2.1. Plant Material

Aerial parts of the plant *Moricandia sinaica* (Boiss) were collected from the region of Hfr-Al-Batin, Saudi Arabia in March-April 2018 and identified by a taxonomist at the Herbarium Unit. Specimens were kept at the herbarium of College of Pharmacy at King Saud University, Riyadh, Saudi Arabia under the code number “SY284”.

### 2.2. Plant Extraction

*M. sinaica* aerial parts were washed with distilled water and dried in the shade. The powdered aerial dried (830 g) was macerated with 80% (*v/v*) aqueous methanol (MeOH) to obtain the methanol extract (141.8 gm total solid). A part of the extract was concentrated under reduced pressure (Rotavapor® R-300, BÜCHI, Switzerland) till dryness (MOR-1, 36 gm). The rest of the extract was concentrated, suspended in 120 mL of distilled water, sonicated (30 min), and defatted with hexane (600 mL) and then extracted with butanol (500 mL). The butanol and the aqueous fractions were concentrated till dryness and designed as MOR-2 (51 gm) and MOR-3 (63 gm), respectively.

### 2.3. Experimental Animals

In this study, “45 male Wistar rats, weighing between 180 ± 20 g, were used. After randomization into various groups, the rats were acclimatized for a period of 7 days under standard conditions at room temperature (25 ± 3°C) with 12 hr/12 hr light/dark cycles. All the animals were fed under strict hygienic conditions with rodent pellet diet and water ad libitum.” The animal experiment ethics committee approved the study (Approval number: 20–015 National Research Center, Egypt).

### 2.4. Experimental Design

Group I served as the normal control, which received oral distilled water for 14 days, and on the 14th day, they were treated with olive oil (1.5 ml/kg, i.p.). Group II served as a toxic control with CCl_4_ and received oral distilled water for 14 days. On the 14th day, they were treated with CCl_4_ (1.5 ml/kg i.p.) diluted (1 : 1) with olive oil.

Group III served as a positive control group. It received oral methanol extract of Silymarine 10 mg/kg for 14 days and on the 14th day animals received CCl_4_ (1.5 ml/kg i.p.) diluted (1 : 1) with olive oil, 2 hr after administration of the last dose of silymarin. Group VI, V, VI, VII, VIII, and IX received oral distilled water for 14 days, and on the 14th day, they received CCl_4_ (1.5 ml/kg i.p.) diluted (1 : 1) with olive oil. At 48 hr after CCl_4_ intoxication, followed by oral administration of different extracts of *M. sinaica* at the doses of 100 and 200 mg/kg were given to rates at 48 hr after CCl_4_ intoxication. All rats were sacrificed 24 hr after CCl_4_ administration. Just before the sacrifice, blood was collected. “After 24 hr of CCl_4_ injection, blood samples from all the rats were collected from the retro-orbital plexus. Serum was separated by centrifugation at 3000 rpm for 15 minutes and was transferred to a prelabeled appender of tubes for assessment of various biochemical parameters for the cardiac and renal function tests. For cardiac function, biochemical parameters such as lactate dehydrogenase (LDH) and creatinine kinase (CK) were analyzed. For the renal function, the biochemical parameters such as creatinine and uric acid were estimated. Immediately, after blood collection, all animals were sacrificed by “ketamine/xylazine” anesthesia, then, heart and kidney samples were collected, washed with chilled normal saline, followed by processing for biochemical estimations in tissues” [18].

### 2.5. Preparation of Kidney and Heart Homogenate

Collected heart and kidney samples were homogenized in an ice-cold 0.15 M KCl solution using a motor-driven Teflon pestle. Homogenized tissues were treated with ethylenediamine tetraacetic acid (EDTA, pH 7.4) followed by centrifugation at 12000 rpm for 20 minutes. The supernatant was used for the estimation of total protein, NP-SH, and malondialdehyde (MDA).

### 2.6. Biochemical Investigation

#### 2.6.1. Estimation of Biochemical Markers in Heart and Kidney Homogenate

Total protein content [19] Malondialdehyde (MDA) [20] and nonprotein sulfhydryls (NP-SH) [21] were estimated in tissue homogenates by the previously described methods. The estimation of malondialdehyde (MDA) and nonprotein sulfhydryls (NP-SH) were used for oxidative stress. In brief, for MDA, 0.2 mL of tissue sample was separately kept in a different test tube and then incubated at 37°C for one hour and then added to one mL of 10% trichloroacetic acid (TCA) and 1 mL of 0.67% thiobarbituric acid (TBA) and then boiled for five minutes at 95°C. The tube was cooled and then centrifuged. The absorbance of the supernatant was measured at 532 nm. For the estimation of NP-SH, 0.1 mL of the supernatant was suspended in tris buffer, 5–5′-dithiobis-(2 nitrobenzoic acid) (DTNB), and absorbance was measured instantly at 412 nm against blank. The result of both MDA and NP-SH was expressed as nmol/g.

#### 2.6.2. Histopathological Study

The treated animals and their controls were sacrificed by decapitation under light diethyl ether anesthesia. The kidney and heart were removed and fixed in 10% formalin. Fixed tissues were dehydrated, embedded in paraffin wax, and sections of 5 *μ*m thickness were cut. Slides were stained with hematoxylin and eosin for histological examination. The sections were examined under an Olympous light microscope.

### 2.7. Statistical Analysis

The data are expressed as mean ± standard deviation (SD) and were statistically analyzed using the one-way analysis of variance (ANOVA) or Student's *t*-test, followed by Dunnett's multiple comparison tests. Statistical significance was set at *p* < 0.05, or *p* < 0.01, or *p* < 0.001.

## 3. Results

### 3.1. Effect of Different Extracts of M. sinaica on Cardiac Function Markers in Serum

Table 1 shows the effects of different extracts of *M. sinaica* on cardiac function markers in CCl_4_-intoxicated rats. LDH and creatinine kinase were significantly (*p* < 0.001) elevated in the CCl_4_ intoxicated rats (190.03 ± 8.89 and 401.50 ± 7.01 mg/dl, respectively) when compared to the normal animals (96.86 ± 3.77 and 208.33 ± 3.91 mg/dl, respectively). Administration of the butanol extract (Mor-2) at doses of 100 and 200 mg/kg prior to CCl_4_ treatment, significantly (*p* < 0.05 − 0.001) protected the elevated LDH and creatinine kinase levels.

### 3.2. Effect of Different Extracts of M. sinaica on Kidney Function Markers

Table 2 shows the effect of different extracts of *M. sinaica* on renal function markers in the CCl_4_-intoxicated rats. The kidney function markers such as creatinine and uric acid in CCl_4_ intoxicated group of rats were 4.10 ± 0.08 and 4.45 ± 0.21 mg/dl, respectively when compare to the normal control group 1.45 ± 0.03 and 1.26 ± 0.08, respectively. The elevated level of renal function markers was significantly (*p* < 0.05 − 0.001) maintained in the butane extract (Mor-2) and silymarin groups of animals (Table 2).

### 3.3. Effect of Different Extracts of M. sinaica on Myocardial Oxidative Stress Markers

Total protein, MDA, and NPSH (oxidative stress profile) of heart tissues were shown in Figures 1–3. The level of total protein (Figure 1) in CCl_4_ intoxicated rats was significantly decreased (*p* < 0.001) when compared to the normal group. The level of total proteins in the butanol extract (Mor-2) (100 and 200 mg/kg) and silymarin (10 mg/kg) groups showed a significant (*p* < 0.05 − 0.001) improvement in the total protein level. The MDA (≈6.59 nmol/g) was elevated in the CCl_4_ intoxicated group when compared to that of the normal group (≈1.11 nmol/g) of rat cardiac tissue (*p* < 0.001). The significant (*p* < 0.05 − 0.001) protective level of MDA (Figure 2) was shown in the butanol extract (100 and 200 mg/kg) and silymarin (10 mg/kg) groups.

Figure 3 showed that NP-SH (≈3.32 nmol/g) level in CCl_4_ was significantly (*p* < 0.001) decreased in comparison to the normal (≈6.30 nmol/g) groups of the rats. Whereas, treatment with the butanol extract (100 and 200 mg/kg) and silymarin significantly (*p* < 0.05 − 0.001) protect the heart tissues.

### 3.4. Effect of Different Extracts of M. sinaica on Renal Oxidative Stress Markers

Total protein, MDA, and NPSH (oxidative stress profile) of kidney tissues were shown in Figures 4–6. The level of total protein (≈43.51) Figure 4, in CCl_4_ intoxicated group was significantly decreased (*p* < 0.001) when compared to the normal control group (≈114.57). The level of total proteins in the butanol extract (100 and 200 mg/kg) and silymarin treated groups showed a significant (*p* < 0.05 − 0.001) protection. The MDA level (≈5.59 nmol/g) was significantly (*p* < 0.001) elevated in the CCl_4_ intoxicated group when compared with the normal control group (≈0.74 nmol/g). The significant (*p* < 0.05 − 0.001) protctive level of MDA (Figure 5) in kidney tissues was shown in the butanol extract (100 and 200 mg/kg) and silymarin (≈2.80, ≈1.92 and ≈1.35 nmol/g, respectively) groups. NP-SH (≈3.29 nmol/g) level (Figure 6) was significantly (*p* < 0.001) decreased in CCl_4_ intoxication when compare to the normal control rats (≈5.72 nmol/g).

Whereas, treatment with the butanol extract (Mor-2) with higher dose and silymarin (≈4.32 and ≈4.97 nmol/g, respectively) significantly (*p* < 0.001) protected the kidney tissues.

### 3.5. Histopathological Results

#### 3.5.1. Kidney

Microscopic investigation of healthy control showed the normal structure of the renal corpuscles and tubules (Figure 7(a)). In the histopathological examination of the injection of CCl_4_, the observed changes showed severe destruction in the curricular region of the kidneys. The damages induced were in the forms of glomerular atrophy disappearance of Bowmen's space, congestion in the capillary loops, and dilation in renal tubules that associated with detachments of their epithelial cell, and foamy look of epithelial cells (Figure 7(b)).

Administration of CCl_4_ along with silymarin revealed the normal feature of the cortex appeared more or less like normal one (Figure 7(c)). On the other hand, some rats of this group showed degeneration of some renal tubules (Figure 7(d)). In case of rats that were given CCl_4_ and MOR-1–100 mg/kg, the glomeruli and many of renal tubules appeared more or less like normal. Degeneration of some renal tubules was noticed (Figure 7(e)). Rats that were administered CCl_4_ and MOR-1 (200 mg/kg) showed that glomeruli and many of the renal tubules appeared normal. But some renal tubules showed mild degeneration of (Figure 7(f)).

Sections of the cortex of the kidney from rats that were treated with CCl4 and MOR-2-100 mg/kg showed the normal structure of renal corpacells and tubules (Figure 8(a)). Nevertheless, CCl4 and MOR-2 (200 mg/kg) exhibited the disturbance of cortex structure that appeared as moderate degeneration of both renal glomeruli and tubules (Figure 8(b)). In the group of CCl4 and MOR-3 (100 mg/kg), the feature of the cortex appeared more or less like the normal one (Figure 8(c)). In contrast, CCl4 and MOR-3-200 mg/kg administered rats showed severe degeneration of some renal glomeruli and tubules (Figure 8(d)).

#### 3.5.2. Heart

Histological examination of sections of the heart from control rats shows the normal structure of myocytes with striations and branched appearance (Figure 9(a)), CCl_4_ administered rats show focal necrosis of muscle fibers with eosinophilia in the cytoplasm. Severe degeneration of the myocytes and congestion of blood vessels (Figure 9(b)), CCl_4_ and silymarin administered rats show the myocytes that appeared more or less like the control one (Figure 9(c)), CCl_4_ and MOR-1 (100 mg/kg) administered rats show the myocytes appeared more or less like the normal one. Notice the degeneration of few myocytes (Figures 9(d)) and 9(e)), CCl_4,_ and MOR-1 (200 mg/kg) administered rats show the myocytes appeared more or less like the normal one (Figure 9(e)).

Longitudinal sections of hearts from rats the CCl4 and MOR-2 (100 mg/kg) showed the normal structure of myocytes (Figure 10(a)). On the other hand, rats of CCl4 and MOR-2 (200 mg/kg) group showed the normal structure of myocytes that were associated with congestion of blood vessels (Figure 10(b)). Heart from rats given CCl4 and MOR-3 (100 mg/kg) showed that the tissue appeared more or less like the normal one (Figure 10(c)). In some rats, CCl4 and MOR-3 (100 mg/kg) group showed the disturbance feature of myocytes and blood vessel congestion (Figure 10(d)). Administration of CCl4 and MOR-3 (200 mg/kg) exhibited the normal structure of myocytes (Figure 10(e)). While in some rats, CCl4 and MOR-3 (200 mg/kg) showed degeneration of some myocytes (Figure 10(f)).

## 4. Discussion

*M. sinaica* is a herbaceous plant, its biological potential, like cardioprotective and nephroprotective, is mostly unexplored. Nevertheless, the therapeutic potential of *Moricandia* genus is in complete agreement with this study. Species of Moricandia genus showed antioxidant, anticancer, antiinflammatory, cytotoxicity, antibacterial, antipyretic, and analgesic activity [22]. Our previous findings showed that *Moricandia sinaica* is rich in phenols, polyphenols, flavonoids, and flavonoid glycosides [19]. The species associated with this genus are traditionally used for pain and syphilis treatment [19]. The present study showed a cardioprotective as well as nephroprotective effect of the butanol fraction of *Moricandia sinaica* herbs. Free radicals increase oxidative stress, which is well recognized in several models of tissue toxicity [23]. Carbon tetrachloride (CCl_4_), a typical toxic agent, produces toxic effects by the production of free radicals (methyl trichloride radicals (CCl_3_^*∗*^)) by the activation of liver cytochrome P450 enzymes [24]. While the liver is considered to be the primary target of CCl_4_ toxicity, it also causes free radical generation in the heart and kidneys [2, 5]. Chloroform and lipid radicals are produced due to the formation of a covalent bond with the unsaturated fatty acids after exposure to CCl4 [25]. The dramatic change of the biological membrane in result of lipids peroxidation, causes a significant role in the different ailments [26]. The findings of the present study showed that injection of CCl_4_ to rats induced oxidative heart damage, which is proved by an increase in the LDH and creatine kinase (ATP restoration enzyme) and decreased albumin levels. The findings of the present study are in agreement with the previous recognition of cardiac damage, which involves the measurements of several cardiac marker enzymes, including lactate dehydrogenase (LDH) and creatinine kinase (CK) [5]. Decreased activities of enzymes in heart tissue and increasing concentration in the serum as an indicator of heart injury [27]. The present finding also showed an increase in malondialdehyde (MDA) and a decrease in the total protein level in hearts of CCl_4_-treated rats when compared with normal rats, showing that the heart is one of the target organs affected by CCl_4_-toxicity. These findings are in agreement with earlier experiments that showed CCl_4_ can cause oxidative damage and produce reactive oxygen species (ROS) in different organs, including the heart [28]. The same is said for several models of nephrotoxicity considering the increased oxidative stress and decrease in antioxidants. CCl_4_ is a well-established model to induce hepatotoxicity and can also be applied to nephrotoxicity by the production of free radicals [29]. In the present study, administration of CCl4 to rats induced oxidative kidney damage, confirmed by an elevation in serum levels of creatinine, uric acid, Na, K, and Ca. According to previous findings, these pathological changes revealed potential damage to kidney cells [30]. The present finding also showed a decrease in total protein, NP-SH and an increased in malondialdehyde (MDA) levels in the kidney tissues of CCl4-treated rats when compared with normal rats. These findings are in agreement with earlier experiments showing oxidative damage and ROS produced by CCl_4_ are responsible for nephrotoxicity [31]. The defensive effects of MOR-2 may be due to protective effects against CCl_4_ causing oxidative stress [32]. Microscopic structural changes in the cardiac and renal tissues of CCl4-intoxicated rats were prevented by pretreatment with MOR-2 in the experimental groups. The significant prevention of the structural alterations indicated that MOR-2 scavenged the free radicals to reduce cellular damage. To find out exactly what the active Phyto-constituent is and its mechanism of action are still required. From those findings' further investigation of the butanol fraction of *Moricandia sinaica* as a cardioprotective and nephroprotective against oxidative radical stress will be of great interest.

## 5. Conclusion

The current finding confirmed that the *Moricandia sinaica* at high doses showed significant cardiac and renal protective activities. Therefore, the plant species *Moricandia sinaica* are highly recommended for the researchers to further explore for isolation of bioactive constituents.

## Figures and Tables

**Figure 1:** Effect of extract fraction on total protein in heart tissue. All values represent mean ± SEM. ^*∗*^*p* < 0.05^*∗∗∗*^*p* < 0.001; ANOVA, followed by Dunnett's multiple comparison test. Where ^a^ compared to the normal group and ^b^ compared with ^a^ groups. I Normal, II CCl_4_, III-Silymarin + CCl_4_, IV-MOR-1 (100 mg/kg) + CCl_4_, V-MOR-1 (200 mg/kg) + CCl_4_, VI-MOR-2 (100 mg/kg) + CCl_4_, VII-MOR- 2 (200 mg/kg) + CCl_4_, VIII-MOR-3 (100 mg/kg) + CCl_4_ and IX-MOR-3 (200 mg/kg) + CCl_4_.

**Figure 2:** Effect of extract fraction on MDA (Malondialdehyde) in heart tissue. All values represent mean ± SEM. ^*∗*^*p* < 0.05^*∗∗∗*^*p* < 0.001; ANOVA, followed by Dunnett's multiple comparison test. Where ^a^ compared to the normal group and ^b^ compared with ^a^ groups. I Normal, II CCl_4_, III-Silymarin + CCl_4_, IV-MOR-1 (100 mg/kg) + CCl_4_, V-MOR-1 (200 mg/kg) + CCl_4_, VI-MOR-2 (100 mg/kg) + CCl_4_, VII-MOR-2 (200 mg/kg) + CCl_4_, VIII-MOR-3 (100 mg/kg) + CCl_4_ and IX-MOR-3 (200 mg/kg) + CCl_4_.

**Figure 3:** Effect of extract fraction on NP-SH (nonprotein and sulfhydryls) in heart tissue. All values represent mean ± SEM. ^*∗*^*p* < 0.05^*∗∗∗*^*p* < 0.001; ANOVA, followed by Dunnett's multiple comparison test. Where ^a^ compared to the normal group and ^b^ compared with ^a^ groups. I Normal, II CCl_4_, III-Silymarin + CCl_4_, IV-MOR-1 (100 mg/kg) + CCl_4_, V-MOR-1 (200 mg/kg) + CCl_4_, VI-MOR-2 (100 mg/kg) + CCl_4_, VII-MOR-2 (200 mg/kg) + CCl_4_, VIII-MOR-3 (100 mg/kg) + CCl_4_ and IX-MOR-3 (200 mg/kg) + CCl_4_.

**Figure 4:** Effect of extract fraction on total protein in kidney tissue. All values represent mean ± SEM. ^*∗*^*p* < 0.05^*∗∗∗*^*p* < 0.001; ANOVA, followed by Dunnett′s multiple comparison test. Where ^a^ compared to the normal group and ^b^ compared with ^a^ groups. I Normal, II CCl_4_, III-Silymarin + CCl_4_, IV-MOR-1 (100 mg/kg) + CCl_4_, V-MOR-1 (200 mg/kg) + CCl_4_, VI-MOR-2 (100 mg/kg) + CCl_4_, VII-MOR-2 (200 mg/kg) + CCl_4_, VIII-MOR-3 (100 mg/kg) + CCl_4_ and IX-MOR-3 (200 mg/kg) + CCl_4_.

**Figure 5:** Effect of extract fraction on MDA (Malondialdehyde) in kidney tissue. All values represent mean ± SEM. ^*∗*^*p* < 0.05^*∗∗∗*^*p* < 0.001; ANOVA, followed by Dunnett's multiple comparison test. Where ^a^ compared to the normal group and ^b^ compared with ^a^ groups. I Normal, II CCl_4_, III-Silymarin + CCl_4_, IV-MOR-1 (100 mg/kg) + CCl_4_, V-MOR-1 (200 mg/kg) + CCl_4_, VI-MOR-2 (100 mg/kg) + CCl_4_, VII-MOR-2 (200 mg/kg) + CCl_4_, VIII-MOR-3 (100 mg/kg) + CCl_4_ and IX-MOR-3 (200 mg/kg) + CCl_4_.

**Figure 6:** Effect of extract fraction on NP-SH (nonprotein and sulfhydryls) in kidney tissue. All values represent mean ± SEM. ^*∗*^*p* < 0.05^*∗∗∗*^*p* < 0.001; ANOVA, followed by Dunnett's multiple comparison test. Where ^a^ compared to the normal group and ^b^ compared with ^a^ groups. I Normal, II CCl_4_, III-Silymarin + CCl_4_, IV-MOR-1 (100 mg/kg) + CCl_4_, V-MOR-1 (200 mg/kg) + CCl_4_, VI-MOR-2 (100 mg/kg) + CCl_4_, VII-MOR-2 (200 mg/kg) + CCl_4_, VIII-MOR-3 (100 mg/kg) + CCl_4_ and IX-MOR-3 (200 mg/kg) + CCl_4_.

**Figure 7:** Sections of the cortex of the kidney from (A-F). (a) control rat shows the normal structure of renal corbacells and tubules (b) rat administered with CCl_4_ onlet show the disturbance of cortex structure. Severe degenerations of both renal glomeruli and tubules are appeared, (c) rat giving CCl_4_ and silymarin administered show the cortex appeared more or less like normal one, (d) rat administered CCl_4_ and silymarin show degeneration of some renal tubules, (e) rat administered CCl_4_ and MOR-1 (100 mg/kg) show the glomeruli and many of renal tubules appeared normal. Notice the degeneration of some renal tubules, (f) CCl_4_ and MOR-1 (200 mg/kg) administered rat show the glomeruli and many of renal tubules appear normal. Notice the degeneration of some renal tubules (H & E stain, Scale bar 5 *μ*m).

**Figure 8:** Sections of the cortex of the kidney from (A-D). (a) CCl_4_ and MOR-2 (100 mg/kg) rat shows the normal structure of renal corpacells and tubules (b) CCl_4_ and MOR-2 (200 mg/kg) administered rat shows the disturbance of cortex structure. Moderate degeneration of both renal glomeruli and tubules appear, (c) CCl_4_ and MOR-3 (100 mg/kg) administered rat show the feature of cortex appeared more or less like the normal one, (d) CCl_4_ and MOR-3 (200 mg/kg) administered rat show severe degeneration of some renal glomerulus and tubules (H & E stain, Scale bar 5 *μ*m).

**Figure 9:** Sections of heart from (A-E). (a) control rat shows the normal structure of myocytes with striations and branched appearance, (b) CCl_4_ administered rat show focal necrosis of muscle fibers with eosinophilia in the cytoplasm. Severe degeneration of the myocytes and congestion of blood vessels, (c) CCl_4_ and silymarin administered rat show the myocytes that appeared more or less like the control one, (d) CCl_4_ and MOR-1 (100 mg/kg) administered rat shows the myocytes appeared more or less like the normal. Notice the degeneration of few myocytes, (e) CCl_4_ and MOR-1 (200 mg/kg) administered rat shows the myocytes appeared more or less like the normal (H & E stain, Scale bar 5 *μ*m).

**Figure 10:** Sections of heart from (A-F). (a) CCl_4_ and MOR-2 (100 mg/kg) rat shows the normal structure of myocytes, (b) CCl_4_ and MOR-2 (200 mg/kg) administered rat shows the normal structure of myocytes that associated with congestion of blood vessels, (c) CCl_4_ and MOR-3 (100 mg/kg) administered rat show the feature of heart tissue appeared more or less like normal one, (d) CCl_4_ and MOR-3 (100 mg/kg) administered rat show the disturbance feature of myocytes and blood vessels congestion, (e) CCl_4_ and MOR-3 (200 mg/kg) administered rat show normal structure of myocytes, (f) CCl_4_ and MOR-3 (200 mg/kg) administered rat show degeneration of some myocytes (H & E stain, Scale bar 5 *μ*m).

**Table 1:** Effect of extracts on Cardiac function test treated with CCl4.

Treatments	Dose (mg/kg0)	Creatine-kinase (mg/dl)		LDH (mg/dl)	
		Mean ± S.E	(%) change	Mean ± S.E	(%) change
Normal		208.33 ± 3.91		96.86 ± 3.77	
CCl_4_		401.50 ± 7.01^*∗∗∗*^	93↑	190.03 ± 8.89^*∗∗∗*^	96↑
Silymarin + CCl_4_	10	234.83 ± 3.74^*∗∗∗*^	42↓	119.60 ± 3.73^*∗∗∗*^	37↓
MOR-1 + CCl_4_	**100**	399.50 ± 4.51		186.37 ± 5.21	
MOR-1 + CCl_4_	**200**	381.00 ± 4.69^*∗*^	5↓	168.81 ± 4.70	11↓
MOR-2 + CCl_4_	**100**	328.66 ± 13.81^*∗∗∗*^	18↓	137.45 ± 4.85^*∗∗∗*^	28↓
MOR-2 + CCl_4_	**200**	269.83 ± 7.50^*∗∗∗*^	32.79↓	127.61 ± 3.60^*∗∗∗*^	33↓
MOR-3 + CCl_4_	**100**	418.16 ± 14.96	4↑	194.95 ± 5.54	
MOR-3 + CCl_4_	**200**	429.00 ± 7.18^*∗*^	7↑	180.50 ± 7.84	5↑

All values represent mean ± SEM. ^*∗*^*p* < 0.05; ^*∗∗∗*^*p* < 0.001; ANOVA, followed by Dunnett′s multiple comparison test. 1-CCl_4_ group compared to the normal group, 2-Treated groups compared with the CCl_4_ group. Bold values are the quantity of dose in mg/kg.

**Table 2:** Effect of extracts on kidney function test treated with CCl_4_.

Treatments	Dose (mg/kg)	Creatinine (mg/dl)		Uric acid (mg/dl)	
		Mean ± S.E	(%) change	Mean ± S.E	(%) change
Normal		1.45 ± 0.03		1.26 ± 0.08	
CCl_4_		4.10 ± 0.08^*∗∗∗*^	181↑	4.45 ± 0.21^*∗∗∗*^	253↑
Silymarin + CCl_4_	10	1.87 ± 0.10^*∗∗∗*^	54↓	1.83 ± 0.08^*∗∗∗*^	59↓
MOR-1 + CCl_4_	**100**	3.81 ± 0.14	7↓	4.59 ± 0.015	3↓
MOR-1 + CCl_4_	**200**	3.09 ± 0.07^*∗∗∗*^	25↓	4.26 ± 0.11	4↓
MOR-2 + CCl_4_	**100**	2.46 ± 0.05^*∗∗∗*^	40↓	3.14 ± 0.19^*∗∗*^	29↓
MOR-2 + CCl_4_	**200**	2.05 ± 0.04^*∗∗∗*^	50↓	2.40 ± 0.11^*∗∗∗*^	46↓
MOR-3 + CCl_4_	**100**	3.80 ± 0.11	7↓	4.50 ± 0.21	
MOR-3 + CCl_4_	**200**	3.12 ± 0.06^*∗∗∗*^	24↓	4.78 ± 0.17	7↑

All values represent mean ± SEM. ^*∗∗*^*p* < 0.01; ^*∗∗∗*^*p* < 0.001; ANOVA, followed by the Dunnett's multiple comparison test. 1- CCl_4_ group compared to the normal group, 2-Treated groups compared with the CCl_4_ group. It is quantity level of doses in (mg/kg).

## Data Availability

All the data are presented in the MS.

## Abbreviations

ANOVA: Analysis of variance
CK: Creatinine kinase
CCl4: Carbon tetrachloride
LDH: Lactate dehydrogenase
MDA: Malondialdehyde
SD: Standard deviation
NPSH: Nonprotein sulfhydryls
MOR-1: Methanol extract
MOR-2: Butanol fraction
MOR-3: Aqueous fraction.
